RETRACTED

# Rehabilitation Treatment of Muscle Strain in Athlete Training under Intelligent Intervention

**DOI:** 10.1155/2022/5403681

**Published:** 2022-03-29

**Authors:** Yu Qiao, Lei Zhang, Bin Zhang

**Affiliations:** ^1^Angeles University Foundation, Angeles City, Pampanga, Philippines; ^2^Anhui Wannan Medical College, Wuhu, 241000 Anhui, China; ^3^Wanjiang College of Anhui Normal University, Wuhu, 241000 Anhui, China

## Abstract

With the development of artificial intelligence technology in the medical field, clinical trials using artificial intelligence as an intervention method are constantly emerging. This article mainly introduces the intervention of artificial intelligence and emotional intelligence on the rehabilitation of athletes' muscle strains. Among them, artificial intelligence and emotional intelligence are a brand-new nursing intervention method. This article compares conventional rehabilitation therapy with these two new types of intelligent interventions to explore the effects of artificial intelligence intervention and emotional intelligence intervention in the rehabilitation of athletes. The experimental results show that the average number of muscle restrains under the intervention of artificial intelligence is 4.1 times, the average restrain rate of muscles is 27.7%, and the average recovery degree of athletes is 94.7%. The average SPB score under emotional intelligence intervention was 56 points. Artificial intelligence interventions can enhance rehabilitation through advanced technology, and emotional intelligence interventions can provide emotional support to effectively improve treatment outcomes and quality of life.

## 1. Introduction

Artificial intelligence technology originated in the 1950s. Artificial intelligence is based on big data network resources. According to the characteristics of human intelligence, the artificial system is simulated and designed with computer information technology using it for the development of machines, software, or new technologies and finally applying them in various fields. With the rapid development of computer technology and the updating of algorithms, artificial intelligence technology has also gone from concept to practical application. It has gradually realized a variety of technologies such as speech recognition, image recognition, language recognition, and natural language processing and is gradually being widely used in education, medical, security, finance, autonomous driving, etc. With the continuous development and maturity of artificial intelligence technology, based on cloud computing, cloud storage, wireless communication, RFID, and other technologies, artificial intelligence technology has been widely used in the medical and health fields. Smart medical refers to a regional medical information platform for establishing medical and health files. It uses artificial intelligence technology to enable patients, medical staff, medical institutions, and medical equipment to communicate with each other and gradually realize information and intelligence. This promotes the development of medical services [1, 2].

RETRACTED

In normal training and high-intensity competitions, athletes often experience sports injuries, which seriously affect athletes' daily training and life. In sports and training, muscle strain is a relatively common sports injury. If too much tension is exerted on the muscle during exercise, it will exceed its capacity. Or the muscles are suddenly stretched too much, which can cause strains. If the later injury is not handled well, or there is no timely rehabilitation treatment, it will lead to the recovery of the muscle, which will lead to the muscle strain again. Therefore, the correct diagnosis and the development of a reasonable rehabilitation treatment plan are very necessary. Based on the background of the Internet of Things, the intelligent medical treatment can provide an intelligent intervention for the muscle strain in the training of athletes.

This article starts from artificial intelligence and emotional intelligence intervention, using intelligent magnetic resonance technology to accurately diagnose and evaluate muscle strains and to provide active psychological counseling to athletes. It explores the effects of these two interventions on the rehabilitation of muscle strains. So that researchers can better carry out such experiments in the future and promote the application of artificial intelligence and emotional intelligence intervention in medical health.

## 2. Related Work

In terms of theoretical research, domestic and foreign experts and scholars have discussed the application and development prospects of artificial intelligence technology in the field of medicine and have done relevant research on various links and applications of medical intelligence. Based on AmI-MS, Cicotti proposes a new hazard-driven and evidence-based V-model approach to monitor medical conditions and better inform medical decisions for physicians. The problem of unsafe medical devices and nonstandard treatment options is addressed by defining a sequential and consistent exploitation process. The novelty of the approach is the intertwining of risk management and software development activities and the use of case studies to explore quality of care issues [3]. Godinho et al. aim to solve the problem of medical data in communication and storage systems by creating a system that simulates a medical image repository in three steps: an index of sample data sets, a pattern extraction, and a modeling of data studies. The system builds up the model based on a representative time window of the medical data repository and extends it for medical data. In addition, the system has been applied in other studies for medical validation, aiming to evaluate the functionality and extensibility of the explored system [4]. Under the existing deteriorating medical safety big data ecosystem, Zhang and Wang design and construct a safe health big data ecosystem on the Hadoop big data platform. The authors use the Hadoop big data platform to realize centralized storage and analysis of the original data using data synchronization and independent data collection system, so that patients can keep themselves informed of their medical treatment and recovery, and thus provide personalized medical management services for patients [5]. Based on the informatization of medical devices and the use of single-disease medical consumables, Jianghua has built an intelligent clinical path and early warning management system based on medical devices, which ensures the rational use of medical devices. The system will improve the means of supervision so that it can better play the role of fine management. By establishing an intelligent clinical pathway management system and early warning systems for medical devices, it can play a better role in guiding the efficient use of healthcare equipment. This will allow monitoring and control of data for future cost-effective analysis of the treatment of individual diseases [6]. Based on the incremental learning method, Ali et al. have built an intelligent medical platform in the form of dialogue to provide medical guidance and recommendation services. The platform shows 90% knowledge acquisition rate, 80% user satisfaction with the system interaction, and 95% system integration accuracy rate with legacy systems [7]. To study and assess the key influencing variables (and their correlation) on consumer adherence decisions, Liu et al. use a mixed modified multiattribute decision model (MADM) for enhancing and promoting the smart medical terminal to achieve the set expected level in all dimensions and standards. MADM uses an improved VIKOR methodology that uses the INRM and DANP impact weights as a combined weight to figure out how to close the gap and offer the optimum enhancement mechanism to reach the set desired level [8]. Alexander et al. report on recent research findings from McKinsey & Company and discuss the development of artificial intelligence in clinical imaging. The article highlights the progress in its clinical application, the prospects for market adoption, and the obstacles that may be encountered. Artificial intelligence will have a significant influence on the clinical imaging market and, in turn, on the way radiosurgeons operate, enabling faster processing times, more precise resolutions, and reduced tasks [9].

RETRACTED

## 3. Artificial Intelligence and Emotional Intelligence

### 3.1. Artificial Intelligence

Since the Dartmouth Conference in 1956, AI has experienced a history of more than 60 years, from calculative intelligence to perceptual intelligence to sensory intelligence, as shown in Table 1. Calculative intelligence is the prototype of AI and is the foundation of AI development. At present, the focus of AI development at home and abroad is still cognitive intelligence, while sensory intelligence is the superior form of AI and is an important breach in the development of AI [10].

#### 3.1.1. Calculative Intelligence Stage

Computational intelligence is the most basic form of artificial intelligence, enabling it to compute, store, and transmit in a way that humans do [11]. Computers are far faster than humans in terms of storage and computation, and they can state and process large amounts of data quickly. In particular, the whole system has a degree of intelligence based on large deposits and megacomputing. Calculative intelligence performs some tasks through methods such as playing chess and searching the Internet. For example, “IBM's Deep Blue Chess” surpassed human beings in 2006, and Google's search engine can help users find relevant information in “tens of thousands” of pages [12]. Its applications in teaching mainly include fast storage and transmission of massive learning resources and intelligent management of students.

#### 3.1.2. Perceptual Intelligence Stage

Perceptual intelligence is an important phase in the current advances in artificial intelligence. It enables robots to read, distinguish, perceive, and respond as humans do. Currently, the growth of perceptual intelligence has become fairly developed. It mainly uses geometrical patterns, deep learning, and other algorithms to simulate human perception and help people complete their work [13]. Its research scope is very wide, including speech recognition and image recognition, such as Amazon's “Alexa” smart assistant and Google assistant. It can support human-computer interactive voice communication in multiple devices and different languages and provide users with personalized services through voice and text retrieval. Baidu image retrieval uses image recognition technology to achieve real-time retrieval, which greatly meets the needs of users. The application of perceptual intelligence in real life mainly includes intelligent transportation, medical health, modern agriculture, energy supply, logistics sales, as shown in Figure 1.

RETRACTED

#### 3.1.3. Sensory Intelligence Stage

Sensory intelligence is an advanced form of artificial intelligence. It imitates the human ability to think, assimilate, and organize knowledge and it has certain concepts, consciousness, and thoughts [14]. In addition to logical thinking, AI in this period also has various modes of thinking such as figurative thinking and inspired thinking that could help or replace certain human tasks in a comprehensive manner. Sensory intelligence is currently a major part of AI research. Cognitive intelligence is a current emerging area of AI research, and various technology companies are actively conducting research with certain results. For example, AlphaGO, an intelligent educational robot developed by the Hong Kong University of Science and Technology, has a “human-like mind.” Its comprehension, articulation, and intelligence will improve with profound study, and it can offer visualized training and automatic learning.

### 3.2. Emotional Intelligence

American psychologists invented the term “emotional intelligence.” It refers to the individual's ability to perceive, clearly understand, and successfully control the feelings of oneself and others. It uses emotional intelligence to intervene in nursing, fully communicate with patients, help patients improve their emotional ability, overcome negative emotions, and thereby improve their mental state [15].

### 3.3. Smart Technology

#### 3.3.1. Wireless Sensing Technology

Wireless sensor technology is a wireless network composed of a large number of sensor nodes with wireless communication functions in a self-organizing and self-management mode. In the application environment, it can collect the data of the connected objects through the sensing device and then present the result obtained by the application system to the receiver at the other end of the network [16, 17].

Figure 2 shows the architecture of the WSN. The whole system generally consists of sensing units, aggregation units (Gateway), and task management units. After collecting the data from the sensors, the self-organizing network of nodes transmits the acquired data to the aggregation gateway [18, 19]. The convergence gateway then transmits this information to external networks such as UAV, satellite communication network, or the Internet. After that, the data information is transmitted to the remote task management server through the external network, so that the received data can be processed on the remote task management server. Finally, the remote task management server will present the result data after preliminary processing to the user. After the user receives the data from the remote task management node, the data will be processed according to their own needs [20].

RETRACTED

When the WSN is working, the sensor unit is mainly responsible for target tracking, location recognition, forwarding, and storage of other sensor node information. At the same time, it can also perform simple data processing. Sensor nodes can communicate wirelessly to form a self-organizing network and transmit the sensed external information to the sink node through multiple hops. The sink node acts as a bridge to connect the wireless sensor network to the external network with a larger communication range for data conversion and transmission. The sink node receives the data from each sensor node and further analyzes and processes the data. Then, the data is transmitted to the server on the task management node [21]. The task management node is responsible for receiving and storing data in the monitored area and providing visual results to end users through the server, thereby realizing real-time monitoring of the system. A typical wireless sensor network structure means that a large number of sensor nodes are randomly distributed throughout the monitoring area, and the information collected from the monitoring target is transmitted through the neighboring nodes by each sensor node, then, the information is processed and data is fused through a predetermined information, and then sent to the terminal via satellite or wired network.

Sensor nodes usually include four modules: sensors, information processing, wireless communication, and energy supply.  Figure 3 represents the configuration of a sensor node. The main task of the sensor module is to collect data from the monitored area. The A/D conversion module converts the information that cannot be directly processed into digital information that can be directly processed by the chip. As the center of the WSN node, the information processor module controls the total wireless sensor network junction as a whole system. It consists of two parts: calculation and storage, which are responsible for storing and processing sensor data from the sensor module, and for information exchange with the wireless communication module. After the wireless communication module is enabled, communication, coordination, and monitoring can be carried out between various node devices. The main function of the energy supply module is to provide energy for several other modules [22].

According to the nanotope architecture of the WSN, the energy consumed by the nodes for communication can be obtained:

(1) $$\begin{array}{c} E_{rt}\left(i,j\right)=E_{rx}\left(i,j\right)+E_{tx}\left(i,j\right). \end{array}$$

Among them, *E*_rx_(*i*, *j*)  is the energy required for the node to receive a packet with a length of *i* bit, it is used by a node to send a packet of length *i* bits.

RETRACTED

The energy *E*_rx_(*i*, *j*) consumed by the node receiving a packet with a length of i bit can be expressed as

(2) $$\begin{array}{c} E_{\text{rx}}\left(i,j\right)=E_{\text{elec}}\times i. \end{array}$$

In formula (2), *E*_elec_ is the energy required by the node receiving circuit to receive *i* bit data.

The energy *E*_tx_(*i*, *j*) consumed by a node to send a packet with a length of *i* bit can be expressed as

(3) $$\begin{array}{c} E_{tx}\left(i,j\right)=E_{elec}\times i+\varepsilon_{amp}\times i\times j^{r}. \end{array}$$

In formula (3), *E*_elec_ is the energy required by the node sending circuit to send *i* bit data, it is the amplification factor of the power amplifier circuit and related to the distance between two nodes in communication. And *j* is the distance between two nodes in communication.

When *j* ≤ *j*_0_, there are

(4) $$\begin{array}{c} E_{\text{tx}}\left(i,j\right)=E_{\text{elec}}\times i+\varepsilon_{fs}\times i\times j^{2}. \end{array}$$

When *j* > *j*_0_, there are

(5) $$\begin{array}{c} E_{\text{tx}}\left(i,j\right)=E_{\text{elec}}\times i+\varepsilon_{\text{mp}}\times i\times j^{4} \end{array}$$

Incorporating formulas (4) and (5) into equation (1), the energy consumed by a node in the wireless sensor network to forward a packet of length *i* is

(6) $$\begin{array}{c} E_{\text{rt}}\left(i,j\right)=\left\{\begin{array}{cc} E_{\text{elec}}\times i\times 2+\varepsilon_{\text{fs}}\times i\times j^{2} & j\leq j_{0}\\ \;E_{\text{elec}}\times i\times 2+\varepsilon_{\text{mp}}\times i\times {\text{j}}^{4} & j>j_{0} \end{array}\right.. \end{array}$$

#### 3.3.2. GPS Positioning

GPS is a new type of satellite-based navigation technology with all-round three-dimensional positioning and navigation on the ground, ocean, and space. As shown in Figure 4, the system has the characteristics of 24 hour, high accuracy, multifunction, fast positioning, etc. It can provide users around the world with three-dimensional navigation, speed, time, and other applications. GPS has been widely used in military and civilian fields.

GPS positioning refers to the calculation of the change in the time coordinate of the distance between the satellite in high-speed operation and the measurement point through GPS. It first obtains the position of the satellite from the navigation information, and then, the receiver calculates the distance of the carrier. The positioning principle is shown in Figure 5. There are two ranging methods: one is to calculate the time between the satellite and the receiver based on the coded information of the ranging, and the other is to measure the carrier phase based on the phase difference between the GPS satellite and the receiver. Both methods use four or more satellites for observation and then use pseudorange and phase to calculate the position of the carrier. But pseudorange positioning has better real-time performance and higher carrier phase accuracy [23, 24].

RETRACTED

When the satellite sends a false stochastic code, the receiver will transmit the same false stochastic code. After a delay *τ* of propagation distance, the satellite signal reaches the receiver and is processed with the local code. The local code is moved to maximize the correlation. The GPS system uses a multisatellite high-orbit ranging system with distance-based ranging and uses four satellites for simultaneous falsely ranging to obtain the location of the receiver [25, 26].

GPS positioning has errors due to satellite timing parameters, satellite almanac parameters, refracted ambient parameters, antenna phase center deviation, and multipath effects. Positioning errors can be divided into regular systematic errors that can be corrected by humans and unexpected and uncertain random errors. The following errors are mainly analyzed.

#### 3.3.3. Satellite Timing Parameters

The satellite timing parameter is the discrepancy that exists on the satellite ephemeris between the satellite orbit represented in the satellite ephemeris and the real orbit. The orbit error depends on the mathematical model of the orbit calculation, the software, the size of the tracking network used, the distribution of the tracking stations, and the length of the tracking station data observation time.

The following formula is usually used to estimate the influence of satellite orbit error on relative positioning:

(7) $$\begin{array}{c} \frac{1}{10}\frac{d\rho }{\rho }<\frac{dB}{\text{B}}<\frac{1}{4}\frac{d\rho }{\rho }. \end{array}$$

Among them, *ρ* is the radial position of the geometric distance from the satellite to the station; *d* is the satellite ephemeris parameter; *B* is the baseline vector length; dB is the baseline vector measurement error caused by the satellite ephemeris error.

#### 3.3.4. Star Clock Error

Although a high-precision atomic clock is installed on the satellite, there are still problems such as frequency offset and frequency drift in the GPS system. The gap for the difference between the star clock and the GPS norm time difference is called the star clock error. The change of satellite clock can be simulated with a quadratic polynomial:

(8) $$\begin{array}{c} ∆t=a_{0}+a_{1}\left(t-t_{0}\right)+a_{2}{\left(t-t_{0}\right)}^{2}. \end{array}$$

RETRACTED

#### 3.3.5. Ionospheric Delay

When an EMI wave travels thru the ionosphere, its path will curve and change its propagation rate. The delay of the ionosphere caused by the refraction of the ionosphere is the ionospheric delay, and the result can be expressed by the following equation:

(9) $$\begin{array}{c} ∆\rho =\int \left(n-1\right)\text{ds}. \end{array}$$

Among them, *n* is the refractive index of the ionosphere.

The phase refractive index in the atmosphere is

(10) $$\begin{array}{c} n_{\rho }=1-40.28\frac{N_{e}}{f^{2}}. \end{array}$$

The group refractive index is

(11) $$\begin{array}{c} n_{g}=1+40.28\frac{N_{E}}{f^{2}}. \end{array}$$

Therefore, the corresponding propagation path delay is

(12) $$\begin{array}{c} ∆\rho_{\rho }=-40.28\frac{N_{\text{e}}}{f^{2}}, \end{array}$$

(13) $$\begin{array}{c} ∆\rho_{g}=40.28\frac{N_{\varepsilon }}{f^{2}}. \end{array}$$

In order to reduce the influence of the ionosphere, the following measures are usually used in GPS positioning: correction by using dual-frequency observation; correction by using the ionospheric model for single-frequency GPS user receivers; simultaneous observation of the same satellite or group of satellites by two or more receivers; and then the difference of the simultaneous observation values.

In the formula, *f* represents the frequency of the electromagnetic wave, and the total amount of electrons along the propagation path of the electromagnetic wave *N*_*ε*_ is expressed as follows:

(14) $$\begin{array}{c} N_{\varepsilon }=\int N_{e}\text{ds}. \end{array}$$

#### 3.3.6. Tropospheric Delay

Tropospheric delay generally refers to the delayed signal formed by the refraction of electromagnetic waves in the troposphere. Because the troposphere is not a dispersive medium for the propagation of electromagnetic waves. That is to say, the tropospheric delay has nothing to do with the frequency of the radio wave, and the dual-frequency correction method cannot be used to reduce its influence, and the model method can only be used [27]. The commonly used tropospheric delay model is the Hopfield model, and the model uses the following formula.

The latency of the dry Tropospheric Fraction in the Zeppo orientation is

(15) $$\begin{array}{c} ∆D_{z,\text{dry}}=10^{-6}k_{1}\frac{P_{s}}{T_{s}}\frac{H_{d}-h}{5}. \end{array}$$

The latency of the wet Tropospheric Fraction in the Zeppo orientation is

(16) $$\begin{array}{c} ∆D_{z,\text{wet}}=10^{-6}\left[k_{3}+273\left(k_{2}-k_{1}\right)\right]\frac{e_{s}}{T_{s}^{2}}\frac{H_{w}-h}{5}. \end{array}$$

Among them, the top heights of the dry and wet atmospheres are

(17) $$\begin{array}{c} H_{d}=40136+148.72\left(T_{s}-273.15\right)\text{m}, \end{array}$$

(18) $$\begin{array}{c} H_{w}=11000\text{m}. \end{array}$$

Therefore, the total tropospheric delay of the zenith is obtained as

(19) $$\begin{array}{c} ∆D_{z,\text{trop}}=∆D_{z,\text{dry}}+∆D_{z,\text{wet}}. \end{array}$$

The projection function of the wet and dry components with the following equation can be stated as

(20) $$\begin{array}{c} M_{\text{dry}}\left(E\right)=\frac{1}{\sin{\left[E^{2}+{\left(2.5^{0}\right)}^{2}\right]}^{1/2}}, \end{array}$$

(21) $$\begin{array}{c} M_{\text{wet}}\left(E\right)=\frac{1}{\sin{\left[E^{2}+{\left(1.5^{0}\right)}^{2}\right]}^{1/2}}.. \end{array}$$

RETRACTED

## 4. System Verification

In the wave of deep learning, technologies such as visual recognition, speech processing, and natural language processing have all made huge breakthroughs. Artificial intelligence has gradually been widely used in the field of healthcare, and its focus is on medical and health management, medical services, rehabilitation, clinical scientific research, and drug development industry management.  Table 2 shows the market size of artificial intelligence in the medical and health field.

In the context of the Internet of Things, the concept of smart medical treatment has emerged. Intelligent medical equipment is combined with modern artificial intelligence technology to perform intelligent diagnosis on medical data. In the field of treatment, surgical robots are used to perform intelligent treatment and to manage big data and normal health services. At the same time, it promotes humanized medical care and allows patients, hospitals, and doctors to communicate closely with each other. Finally, patients can achieve disease prevention and treatment.  Figure 6 shows the smart medical structure diagram.

The wide utilization of AI technique in healthcare not only solves people's urgent needs for health but also promotes the integration and optimization of the entire medical industry. The rapid development of medical technology can intelligently analyze the patient's body data, synchronize medical, equipment, drug and other data, and process and update them in a timely manner. In this way, the core services of the medical platform can be improved and medical safety risks can be minimized. Currently, with the increasing innovation of IOT, Da Data, cloud computing, the intelligent sanitation management industry, and equipment have achieved rapid development. At home, people can use the Internet and medical equipment to seek medical treatment, check their health in a timely and convenient manner, and conduct disease prevention and early diagnosis. The intelligent medical Internet of Things solves the technical bottleneck and makes the health management model gradually enter the lives of ordinary people. With the user's health file as the core, through the integration of information technology, a medical and health service platform with the patient's health file as the core is established. Intelligent collection of patient data can enable better configuration of regional medical and health services and can also reduce risks in the medical process, allowing patients to enjoy better medical services under convenient and fast conditions.

RETRACTED

The use of AI in the health care arena can be divided into three processes. The first process is medical informatization, that is, through various network technologies, medical data and information can be presented on multiple platforms; the second process is medical networking. Through RFID technology, Wind computing, Da Data, and other technologies, various links of network consultation, hospital visits, and postdiagnosis observation can be implemented smoothly, and medical accuracy and efficiency can be improved; the third process is intelligent medical treatment. It uses artificial intelligence machine learning and calculation methods for intelligent diagnosis, surgical robots for intelligent treatment, medical databases for tracking and analysis of cases, and electronic medical assistants to assist doctors in treatment. Realizing the intellectualization of the whole process of medical treatment and health care runs through the whole medical treatment. It includes disease prevention and health management before diagnosis, auxiliary diagnosis during diagnosis, clinical decision making, auxiliary post-diagnosis treatment and other auxiliary rehabilitation. At present, the adoption of AI in the healthcare arena in China is still in the second stage, but it is moving towards the third stage.

## 5. Experimental Design of Athlete Muscle Strain Rehabilitation

In order to observe the clinical effects of the middle and late rehabilitation treatment of muscle strains, three different treatment programs were performed on muscle strain patients during the muscle strain period, and the treatment effects and the incidence of restrains of the three groups of patients were observed.

Thirty cases of athletes with muscle strains, aged 18-24 years, were randomly chosen as study subjects. The athletes were split arbitrarily among reference team, experimental team 1, and experimental team 2, with 10 cases in each team. There was no apparent statistical difference in the strains among the three groups, and they were comparable.

RETRACTED

The reference team received traditional muscle exercise rehabilitation treatment. And the specific methods were as follows: after 2 to 3 days of injury, perform restorative exercise on the injured part of the athlete. Under the protection of elastic bandages, first perform static training, then transition to dynamic training, and finally speed training. The best practice intensity is to reduce static training: Use exercises such as thigh tightening, calf tightening, and static resistance to statically contract the muscles for 5 to 10 seconds, with an interval of 10 to 20 seconds. Repeat the exercise 10 times, 1 to 2 times a day. Dynamic training: muscle contraction through exercises such as supine leg lift or prone straight leg, heel lift, and squat-up exercises. When the muscle is contracted to its maximum amplitude, keep it for 3 ~ 5 s. Repeat the exercise 10 times, 1 to 2 times a day. Speed training: After the athlete's muscles have basically returned to normal, they can start running training and gradually complete the transition from jogging to normal running and fast running.

Experimental team 1 used intelligent magnetic resonance technology to make accurate diagnosis and assessment of muscle strain and then used acupuncture therapy to implement rehabilitation treatment. Specific method: Oblique acupuncture treatment is performed on the injured area with a suitable filigree needle to find the most obvious tenderness point, and puncture the needle about 1 inch above, below, left, and right from the pain point. The needle and the skin form an angle of about 45 degrees, reaching the depth of the injured muscle bundle. The upper and lower needles are treated with an electroacupuncture instrument, with continuous wave treatment for 10 minutes, and then dense wave treatment for 10 minutes. It is once a day, the intervention time is two weeks.

Experimental team 2 added the content of cognitive and emotional intelligence intervention on the basis of conventional rehabilitation treatment. The specific measures are as follows: Adopt the method of diversion, use emotional communication, encourage patients to cultivate positive psychological cues, and enable patients to spontaneously and actively participate in sports exercises; Improve patients' cognitive execution ability and help patients formulate clear rehabilitation goals and daily plans; Enhance patients' awareness of participation, establish tripartite awareness of participation with patients and their families, communicate together, and give patients emotional support. The intervention time is two weeks.

### 5.1. Number and Rate of Muscle Strains

Figure 7(a) is a comparison diagram of the number of muscle strains among the reference team and experimental team 1. The abscissa is different sample cases, each group has 10 cases. The ordinate is the number of muscle strains. The average number of muscle restrains in the control group was 6.7 times, while the average number of muscle restrains in the observation group 1 was 4.1 times.  Figure 7(b) is a comparison diagram of the muscle restrain rate among the reference team and experimental team 1. The abscissa is different sample cases, and the ordinate is the muscle restrain rate. The average restrain rate of muscles in the reference team was 50.1%, while the average restrain rate of muscles in experimental team 1 was 27.7%. As shown in Figure 7, both muscle tone and myotonia were remarkably less in experimental team 1 compared to the reference team. The incidence and prevalence of muscle injuries in the athletes under the artificial intelligence intervention were reduced compared to the conventional method.

RETRACTED

### 5.2. Mental Health Assessment

Mental health assessment of patients. In this study, “self-perceived burden” was assessed as an indicator of “self-perceived burden.” This scale is divided into 10 items with a total score of 100. The higher the score, the higher the psychological stress of the patient and the worse his or her mental state.  Table 3 shows the SPB scores of the control group and the experimental team 2.

Figure 8(a) shows the SPB scores of the control group before and after the intervention, and Figure 8(b) shows the SPB scores of the observation group 2 before and after the intervention. The abscissas and ordinates are the sample and SPB scores, respectively, with an average SPB score of 82 points before intervention. The average SPB score of athletes in the control group was 78 points after the intervention, and the average SPB score of the observation group 2 after the intervention was 56 points. It can be seen from Figure 8 that the self-perceived burden after the intervention is lower and the mental health status is better. The degree of mental health under the intervention of emotional intelligence is significantly better than that of conventional treatment programs.

### 5.3. Life Quality Assessment

The patients' quality of life was assessed to evaluate the quality of survival both preintervention and postintervention. Four quality-of-life rating scales were used, including four items: sensory, motor, self-care, and normal activities. The higher the mark, the greater the improvement in quality of life, as shown in Table 4.

Figure 9(a) shows the evaluation scores of the athletes' quality of life in observation group 1 before and after the intervention, and Figure 9(b) shows the evaluation scores of the athletes' quality of life in observation group 2 before and after the intervention. The abscissa is the sample case, and the ordinate is the quality of life assessment score. The athletes' average quality of life score before intervention was 66.5. The mean quality of life score after the intervention was 82.9 for experimental team 1 and 74.4 for experimental team 2 after the intervention. As shown in Figure 9, the quality of life scores were higher postintervention than preintervention. After the intervention, the score of quality of life was significantly higher in experimental team 1 than in experimental team 2.The quality of life was better in the AI intervention group compared to the emotional intelligence intervention group.

RETRACTED

### 5.4. Degree of Rehabilitation

Figure 10(a) shows the rehabilitation degree of athletes in the reference team and experimental team 1 after intervention, and Figure 10(b) shows the rehabilitation degree of athletes in the reference team and experimental team 2 after intervention. The average rehabilitation degree of the athletes in the reference team was 81.3%, the average rehabilitation degree of the athletes in the experimental team 1 was 94.7%, and the average rehabilitation degree of the athletes in the experimental team 2 was 82.6%. It can be seen from Figure 10 that the average rehabilitation degree of the athletes in reference team 1 is higher than that of reference team 2 and the reference team, and the effect of emotional intelligence intervention on the rehabilitation degree of athletes is not obvious. The average rehabilitation degree under artificial intelligence intervention is higher than the average rehabilitation degree under emotional intelligence intervention.

## 6. Conclusion

The experimental findings have shown that the mean time of muscle restrain under AI intervention was 4.1, and the average restrain rate of muscles is 27.7%, and the average recovery degree of athletes is 94.7%; In the reference team, the average number of muscle restrains was 6.7 times, the average muscle restrain rate was 50.1%, and the average recovery degree of athletes was 81.3%. In contrast to the reference team, the number of muscle strains under the intervention of artificial intelligence was significantly reduced, and the degree of recovery was higher; the mental health under the intervention of emotional intelligence was better. Moreover, under the intervention of artificial intelligence, the quality of life of athletes is better than that under the intervention of emotional intelligence. In summary, artificial intelligence intervention has a significant effect on the promotion of muscle rehabilitation for athletes' muscle strains. At the same time, emotional intelligence intervention can help enhance athletes' mental health and promote muscle recovery. Of course, there are still some shortcomings in this study, the sample size of the experiment is too small, only 30 cases of muscle injury patients were selected, only 10 cases in each group, the sample size can be increased, so that the conclusions drawn are more convincing.

RETRACTED

## Figures and Tables

**Figure 1:** Artificial intelligence application field.

**Figure 2:** Network structure of wireless sensor network.

**Figure 3:** Sensor node structure diagram.

**Figure 4:** GPS positioning system chart.

**Figure 5:** GPS positioning principle diagram.

**Figure 6:** Intelligent medical structure diagram.

**Figure 7:** Diagram of muscle restrain.

**Figure 8:** Self-perceived burden score chart.

**Figure 9:** Quality of life score chart.

**Figure 10:** Rehabilitation degree comparison chart.

**Table 1:** The three stages of artificial intelligence development.

Development stage	Feature	Application
Computing intelligence	Can store and compute	Storage and delivery of massive learning resources and intelligent management system for student information
Perceptual intelligence	Can listen and speak, see, and recognize	Language teaching, oral assessment, and image search
Cognitive intelligence	Can understand and think	Personalized learning and independent learning

**Table 2:** China's artificial intelligence medical market size.

Time	Market size of artificial intelligence in medical field/100 million yuan	Growth rate
2015	120	—
2016	160	0.25
2017	220	0.65
2018	415	0.7
2019	660	0.65
2020	890	0.4

**Table 3:** Self-feeling burden table.

	Before intervention	Control group intervention	Observation group 2 intervention
Sample 1	90	80	70
Sample 2	80	80	60
Sample 3	90	90	60
Sample 4	70	70	50
Sample 5	80	80	60
Sample 6	80	70	50
Sample 7	100	90	60
Sample 8	60	60	40
Sample 9	90	80	60
Sample 10	80	80	50

**Table 4:** Quality of life assessment form.

Quality of life index	Marks
Feeling	25
Body movement	25
Self-care	25
Normal activity	25

## Data Availability

No data were used to support this study.
